# Effects of Mood Regulation on Sociodemographic Status, Exercise Pattern, and Physical Conditions of Chinese Adults and the Elderly

**DOI:** 10.1155/2022/2034957

**Published:** 2022-07-04

**Authors:** Jingjing Lou, Tong Li, Xuefeng Gao, Ying Hu, Xiao Chen, Fan Yang, Xiabing Zheng, Weirui Yang, Liangrong Zheng, Qi Zhu, Yaqi Zhang, Nianhong Guan

**Affiliations:** ^1^Guangzhou Institute of Sports Science, Guangzhou, Guangdong 510620, China; ^2^Department of Psychology, The Third Affiliated Hospital of Sun Yat-sen University, Guangzhou, Guangdong 510630, China; ^3^Tianhe Sports Center, Guangzhou, Guangdong 510620, China

## Abstract

**Objective:**

This study focused on mood regulations and their association with sociodemographic status, exercise pattern, and physical conditions of adults and older adults in China who did not undergo interventions.

**Method:**

Data were based on the 2016 to 2018 Guangdong National Physique Monitoring data, in which 5242 participants aged 20-69 years were recruited. Multiple statistical analysis methods, such as descriptive and logistic regression analyses, were used to study each exercise motivation and its association with influencing factors, including sociodemographic characteristics, exercise measurements, and physical conditions. An exercise index for mental health was also used to investigate the number and types of people who were more likely to meet the index.

**Results:**

We observed that 44.9% (2355/5242) of participants did not engage in physical exercise in this study. Only older participants (40 to 69 years old) and those with an average level of education (high school/technical secondary school) showed a significant association with exercising for mood regulation. Few people met the index that is good for mental health (16.64% [872/5242] met index 1, and 2.84% (149/5242) met index 2), and higher education showed a significant association with a reduction in the mental health burden and the prevention of depression.

**Conclusion:**

This study found that motivating people to be more active and educating them on the potential mental health benefits of exercise could help them to exercise more.

## 1. Introduction

Depression is a common mood disorder affecting individuals of all ages and is characterized by persistent sadness, a loss of interest in activities, energy loss, appetite changes, etc. It is reported that more than 300 million people are now living with depression, which increased by more than 18% between 2005 and 2015 [1]. Its morbidity varies by country and region, but patterns and trends for depressive disorders are remarkably similar worldwide [2]. Depressive disorders can occur comorbidly with nearly every other form of psychopathology in an unsystematic way, leading to greater symptom severity and disability, more attempted suicides, and poorer treatment response [3]. Major depressive disorder, accounting for 4.4% of the disease burden worldwide, increased in rank from the 15th to 11th, for which the cost of the traditional pharmacological treatment could reach approximately US $91 billion in 2030 [4, 5]. Depressive symptoms can significantly decrease the quality of life even if an individual does not meet the threshold for a diagnosis of major depressive disorder [6]. However, depression remains widely undiagnosed and untreated because of stigma, a lack of effective therapies, and inadequate mental health resources [7].

Greater depression is associated with physical inactivity, but evidence suggests that exercise has a large and significant antidepressant effect in people with depression symptoms and in those who are diagnosed with depression [8–10]. Meanwhile, with a large portion of patients with depression who do not properly respond to drug treatment (30% response without remission, 20% partial remission, and 50% remission) [11], exercise is an effective, safe, easily accessible, inexpensive form of therapy that requires less clinician training to perform and carries a low risk of negative side effects [12]. It should be added along with standard drug treatment to improve the health status of patients [13, 14]. Converging evidence suggests that exercise and antidepressant medication may alleviate depression through common neuromolecular mechanisms, including increased expression of neurotrophic factors, increased availability of serotonin and norepinephrine, and reduced systemic inflammatory signaling [15]. In a large US cohort, individuals who exercised had fewer days of poor mental health than those who did not exercise [16]. Regular exercise can protect against future risk of depression in individuals of all ages [17, 18], which was confirmed in a meta-analysis sampling from 105 studies, which highlighted the role of regular aerobic exercise in increasing feelings of well-being and suggested that its absence can have detrimental effects on physical and mental health [19].

Although the benefits of exercise are well described, the high rate of inactivity is worrisome. Recently, it was shown that 31% of adults are physically inactive globally, and physical inactivity is responsible for 6% of deaths globally, making it the fourth-leading risk factor for mortality worldwide [20, 21]. The Active People Survey from Sport England in 2015–2016 found that only 36% of adults reported taking part in sports once a week [22]. The percentage of the population who reported never engaging in moderate physical activity was 66% in Nepal and 64.9% in Bangladesh, based on the WHO World Health Survey [23]. Similarly, people with depression had a high rate of physical inactivity [24]. A total of 34.8% of participants with depression were physically inactive according to data from 24,230 people with depression across 46 low- and middle-income countries [25].

The reasons affecting people's exercise decisions are complex and could include influencing factors such as sociodemographic status, self-efficacy [26], weight loss [27], enjoyment, and physical health [28]. In another review of the salient exercise psychology literature, studies have emphasized that mood regulation depends on interactions among participants, exercise type, and practice conditions and have made several recommendations for structuring an exercise session to maximize mood regulation [29]. Although knowledge of the relationship between exercise and mood regulation is substantial, few studies have investigated the role of specific exercise motivations, especially mood regulation, in relation to sociodemographic status, exercise pattern, and physical condition in the absence of interventions.

This study is aimed at determining the effects of exercises on mood regulation and the reasons affecting peoples' decision to exercise in a nonintervention condition to provide a theoretical and potentially practical basis for future research on exercise interventions.

## 2. Methods

### 2.1. Participants

This study was based on the 2016 to 2018 Guangdong National Physique Monitoring data from the Guangzhou Institute of Sports Science (Guangzhou, China). We measured mental health burden (in this study, mental health burden was considered as a generalized term that could mentally affect the participants due to changes in their physical appearance, behaviors, and daily life if they do not exercise) according to participants' responses to the following question: “what is the main reason why you perform physical exercise?” The answers could be chosen from the following options: (1) disease prevention and treatment, (2) entertainment, (3) mood regulation, (4) losing weight, (5) bodybuilding, (6) social contact, (7) improving motor skills, (8) increasing physical activity, (9) unclear motivation, and (10) other motivation. To study the factors influencing different exercise motivations, missing data for exercise motivation were excluded. Only data from adults (20–59 years) and senior adults (60–69 years) who had clear exercise motivations were used for this study.

### 2.2. Anthropometric Measurement

The participants' height, weight, and abdominal circumference data were obtained from interviewer-administered questionnaires and standardized physical and physiological measurements. Participants were weighed in lightweight clothing without shoes to the nearest 0.1 kg on a calibrated digital scale, and the height was measured to the nearest 0.1 cm with a calibrated stadiometer [30].

Waist circumference measurements were taken horizontally to the nearest 0.1 cm at the midpoint between the inferior margin of the last rib and the iliac crest, with participants standing with feet 25–30 cm apart. Body mass index (BMI) was calculated as weight divided by height squared (kg/m^2^). The World Health Organization (WHO) BMI cutoff points for Asian populations were used to define underweight (BMI < 18.5 kg/m^2^), normal weight (BMI = 18.5–22.9 kg/m^2^), overweight (BMI = 23–24.9 kg/m^2^), obese I (BMI = 25–29.9 kg/m^2^), and obese II (BMI ≥ 30 kg/m^2^) [31]. The WHO recommended the International Diabetes Federation criteria for ethnic- or country-specific values for waist circumference. Waist circumference cutoff points for Chinese individuals were used to define abdominal obesity (waist circumference > 90 cm in men or >80 cm in women) [32].

### 2.3. Covariate Measurement

Sociodemographic characteristics were assessed using the National Physique Monitoring questionnaire. Sociodemographic variables included gender, age, highest education level, and occupations/jobs. For educational background, the participants were classified as having graduated from primary school or below, middle school, high school/technical secondary school, and college/junior college or above. In regard to participants' occupations/jobs, they were classified as students, administrative staff and professionals, business service employees, workers, others, and homemakers and retired individuals.

### 2.4. Measurement of Exercise Characteristics

Exercise characteristics included exercise frequency, exercise duration each time, exercise duration per week, and exercise intensity. All participants were asked “Have you engaged in physical exercise since last year?” The response options were “yes” and “no.” All participants were asked how often they engaged in exercise, with the following seven possible response options: (1) less than once a month, (2) over once a month but less than once a week, (3) once a week, (4) twice a week, (5) three times a week, (6) four times a week, and (7) five times a week or over. Participants were also asked about exercise duration during each exercise session. We estimated exercise duration per week by multiplying exercise frequency by exercise duration each session. Exercise intensity was divided into mild, moderate, and heavy according to changes in respiratory rate, heart rate, and sweating compared to those measured at rest.

### 2.5. Basic Disease Measurement

For basic diseases, participants were asked “Have you ever been diagnosed with the diseases below by experts or doctors?” The response options included the following: (1) hypertension, (2) hyperlipidemia, (3) hypercholesterolemia, (4) diabetes, (5) coronary heart disease, (6) peptic ulcer, (7) osteoarthropathy, and (8) cervical spondylopathy.

### 2.6. Exercise Index for Mental Health

Evidence for the optimal exercise duration of each session (45 min) and exercise frequency (between three and five times per week) was reported to reduce participants' mental health burden [16]. We divided the data into “exercise index for reducing the mental health burden” (exercise 30-60 min each session and 3-5 times per week or over), coded as “meet index 1,” and “exercise index not for reducing the mental health burden” (less than 30 min or more than 60 min per week and less than 3 times per week), coded as “unmet index 1,” according to the recommendation above.

In Samuel's study of “exercise and the prevention of depression,” it was suggested that assuming the relationship is causal; 12% of future cases of depression could have been prevented if all participants had engaged in at least 1 hour of physical activity each week. According to this recommendation, we divided the data into “exercise index for the prevention of depression” (the exercise motivation is mood regulation, and exercise is performed 60-120 min each week), coded as “meet index 2,” and “exercise index not for the prevention of depression” (the exercise motivation is not mood regulation, or exercise is performed less than 60 min or over 120 min each week), coded as “unmet index 2” [17].

### 2.7. Statistical Analysis

All analyses were conducted using SAS 9.4 (SAS Institute Inc., Cary, NC). A *p* value of <0.05 was considered significant.

We used descriptive statistics to report the frequency of sociodemographic characteristics (gender, age, highest education level, and job), exercise measurements (exercise frequency, exercise duration each session, exercise duration per week, and exercise intensity), and physical conditions (BMI, abdominal obesity, and basic diseases). Chi-square tests and *t*-tests were used to compare frequencies data. Disordered multiclassification logistic regression models were used to determine if the observed differences between exercise motivations, mood regulation and sociodemographic characteristics, exercise measurements, and physical condition remained significant. Both the likelihood ratio test and the Wald test were used in the study as well.

We used PROC SURVEYFREQ to calculate prevalence and 95% CIs for the eleven categories of exercise motivations as follows: (1) disease prevention and treatment, (2) entertainment, (3) mood regulation, (4) increasing physical activity, (5) weight loss, (6) social contact, (7) disease prevention and treatment and entertainment, (8) disease prevention and treatment and mood regulation, (9) entertainment and mood regulation, (10) whether the participant has met index 1, and (11) whether the participant has met index 2. A series of multiple logistic regression analyses were conducted to examine the associations of the different exercise motivations listed above with sociodemographic characteristics, exercise measurements, and physical conditions. We reported odds ratios (ORs) with corresponding 95% confidence intervals (95% CIs).

### 2.8. Ethics

The study protocol was approved by the ethical review committee of Guangzhou Institute of Sports Science, Administration of Sports of Guangzhou Municipality. Written informed consent was obtained from each participant at enrollment.

## 3. Results

As shown in Table 1, a total of 5242 participants were involved in this study (47.3% male and 52.7% female). The participants had a high physical inactivity rate of 44.9% (2355/5242). Logistic regression analyses of sociodemographic characteristics, exercise measurements, and physical conditions are shown in Table 2. There were different patterns of characteristics within these 9 categories of exercise motivations.

Regarding the sociodemographic characteristic of gender, there was no significant difference between gender and the exercise motivations of mood regulation, increasing physical activity, weight loss, and social contact. However, men were more likely to exercise for disease prevention and treatment (OR = 1) than women (OR, 0.72; 95% CI, 0.64-0.80), and women were more likely to exercise for entertainment (OR, 1.29; 95% CI, 1.16-1.45, *p* < 0.001) than men. The sociodemographic characteristics of age were significantly associated with each exercise motivation (*p* < 0.001). Interestingly, participants aged 20-29 years old were most likely to exercise for disease prevention and treatment (OR = 1) far more than participants in other age groups. Of 863 participants aged 20-29 years old, 800 (92.7%) had chosen disease prevention and treatment. Participants aged 30-39 years old (OR, 23.03; 95% CI, 17.48-30.34) were most likely to exercise for entertainment. Middle- to older-aged participants (40-49 years old (OR, 1.66; 95% CI, 1.38-1.99), 50-59 years old (OR, 1.78; 95% CI, 1.48-2.14), and 60-69 years old (OR, 1.40; 95% CI, 1.16-1.86) were more likely to exercise for mood regulation. Compared to younger participants, elderly participants (60-69 years old) preferred to exercise for weight loss (OR, 3.65; 95% CI, 2.79-4.77) and social contact (OR, 3.40; 95% CI, 2.33-4.96).

Our results also showed that participants with an education level of college or junior college or above (OR, 0.8; 95% CI, 0.67-0.95) were less likely to exercise for mood regulation than middle- to high-school or technical secondary school educational level participants. With higher education levels, more participants were likely to exercise for disease prevention and treatment. Students (OR = Ref) were most likely to exercise for disease prevention and treatment. Exercise for entertainment seemed more attractive for business service employees (OR, 11.54; 95% CI, 6.27-21.23). Workers (OR, 2.04; 95% CI, 1.29-3.21), administrative staff and professionals (OR, 1.67; 95% CI, 1.08-2.58), homemakers and retired individuals (OR, 1.58; 95% CI, 1.04-2.41), and others (OR, 1.73; 95% CI, 1.12-2.65) were more likely to exercise for mood regulation than students (OR = Ref) and business service employees (OR, 1.14; 95% CI, 0.74-1.75). Homemakers and retired participants were most likely to exercise for weight loss (OR, 4.11; 95% CI, 1.90-8.89).

Exercise characteristics included exercise frequency, exercise duration of each session, exercise duration per week, and exercise intensity. In this study, 44.9% (2355/5242) of participants did not engage in physical exercise. Mood regulation had no significant association with exercise frequency, as did increasing physical activity, weight loss, and social contact. Participants whose exercise motivation was disease prevention and treatment were more likely to exercise less than once a week (OR, 1.37; 95% CI, 1.10-1.71), once a week (OR, 1.41; 95% CI, 1.14-1.73), or over four times a week (OR, 1.22; 95% CI, 1.06-1.41) than they were to engage in no exercise (OR = Ref) and other exercise frequencies. For the motivation of entertainment, participants were more likely to exercise three times weekly (OR, 1.31; 95% CI, 1.05-1.64) and less likely to exercise four times weekly (OR, 0.79; 95% CI, 0.68-0.91) than they were to engage in no exercise (OR = Ref) and other exercise frequencies.

Further, exercise duration for each session or per week showed no significant relationship with mood regulation. For disease prevention and treatment, participants were more likely to exercise less than 30 min (OR, 1.34; 95% CI, 1.07-1.67) and 30-60 min (OR, 1.25; 95% CI, 1.10-1.43) than to engage in no exercise (OR = Ref) and in over 60 min each session (OR, 1.16; 95% CI, 1.00-1.34); they also preferred to exercise 0-30 min (OR, 1.39; 95% CI, 1.14-1.69), 31-60 min (OR, 1.38; 95% CI, 1.11-1.73), and 121-240 min (OR, 1.23; 95% CI, 1.07-1.42) per week than to engage in no exercise (OR = Ref) and other duration of exercise per week.

For the motivation of social contact, fewer people preferred to exercise 30-60 min each session (OR, 0.75; 95% CI, 0.58-0.95) than to engage in no exercise (OR = Ref) and other duration of exercise each session. People who exercise for entertainment were more likely to exercise 61-120 min per week (OR, 1.28; 95% CI, 1.02-1.63) than to engage in no exercise (OR = Ref) and other duration of exercise per week. Participants who exercise to increase physical activity were less likely to exercise 0-30 min per week (OR, 0.72; 95% CI, 0.54-0.97) than to engage in no exercise (OR = Ref) and other duration of exercise per week.

Our findings also showed no significant relationship between exercise intensity, mood regulation, and other exercise motivations, such as entertainment and weight loss. Exercise intensity only showed a significant association between disease prevention and treatment (*p* < 0.001) and social contact (*p* < 0.05). Participants who exercised for the motivation of disease prevention and treatment were more likely to engage in moderate- (OR, 1.22; 95% CI, 1.07-1.39) or heavy-intensity exercise (OR, 1.48; 95% CI, 1.25-1.75). Participants who exercise for social contact were more likely to engage in mild-intensity exercise (OR, 1.35; 95% CI, 1.03-1.78).

Exercise motivations showed no significant association with abdominal obesity (*p* > 0.05) and peptic ulcer (*p* > 0.05), which is why these factors were not listed in Table 2. BMI only had a significant association with disease prevention and treatment, and the underweight participants (OR = Ref) were most likely to choose this motivation. Our research found no significant association between mood regulation and all kinds of diseases. Fewer participants in our study preferred to exercise for disease prevention and treatment with respect to hypertension (OR, 0.65; 95% CI, 0.55-0.77), hyperlipidemia (OR, 0.76; 95% CI, 0.60-0.96), hypercholesterolemia (OR, 0.73; 95% CI, 0.57-0.93), osteoarthropathy (OR, 0.71; 95% CI, 0.57-0.89), and cervical spondylopathy (OR, 0.76; 95% CI, 0.64-0.91). Participants with hypertension preferred to exercise to increase physical activity (OR, 1.35; 95% CI, 1.10-0.65) and lose weight (OR, 1.60; 95% CI, 1.30-1.95).

Concerning indexes 1 and 2, only 16.64% (872/5242) were compliant with index 1, and 2.84% (149/5242) were compliant with index 2. Participants with higher education levels were more likely to meet both indexes 1 and 2 (Table 3). More participants with education levels of college/junior college or above (OR, 3.41; 95% CI, 1.74-6.66) and high/technical secondary school (OR, 2.13; 95% CI, 1.10-4.10) met index 1 than did participants with education levels of middle school (OR, 1.49; 95% CI, 0.77-2.87) and primary or below (OR = Ref). More participants with education levels of college/junior college or above (OR, 2.08; 95% CI, 1.58-2.75) and high/technical secondary school (OR, 1.76; 95% CI, 1.36-2.28) met index 2 than did participants with education levels of middle school (OR, 1.30; 95% CI, 1.00-1.67) and primary school (OR = Ref) (Table 4).

## 4. Discussion

In terms of gender differences in depression, major depression is generally believed to be twice as prevalent among women than in men and represents a major health disparity [33]. In this study, rather than a 2-fold difference, no gender difference was observed among those who exercised for mood regulation. Similar to mood regulation, there was also no gender difference for increasing physical activity, weight loss, and social contact. However, men were more likely than women to exercise for disease prevention and treatment, and women were more likely than men to exercise for entertainment. Female sex was a significant sociodemographic correlate of low physical activity [34, 35]. The rate of no exercise among women was 43.0% (1066/2480), which was lower than the corresponding rate among men (46.7%, 1289/2762, *p* value = 0.007). Generally, women have hobbies that can keep them at home longer than men, while men tend to engage in more outdoor physical recreational activities [36]. Physical activity for leisure was not associated with depression among Brazilian females, and this association was significant among Brazilian males, who might be able to benefit from physical activity for leisure to reduce their symptoms of depression [37].

The reasons why people engage in physical activity might differ among young, middle, and older adults as a result of changing ideologies, life tasks, goals, and health circumstances overtime [38]. The exact manner in which motivation to exercise shifts with increasing age was not fully understood. The motivators of people exercising were proven to shift from future-oriented goals to more present-focused and emotionally meaningful goals as they aged. It was revealed that younger adults prefer to convey expert knowledge of instrumental support, helping to facilitate and engage in challenging workouts, but distinct age-related prioritizations of social factors emerged in motivations to exercise, emphasizing the maintenance and fostering of relationships and increased opportunities for socializing [39]. In our study, young participants in 20-29 years old were most likely to exercise to prevent and treat disease, which was a future-oriented goal. Those between 30 and 39 years of age were most likely to exercise for entertainment as a transition stage, as they had more financial stability than younger participants and fewer worries than older participants related to work stress, depression, illness, obesity, and social requests. Older participants between 40 and 69 years were more likely than younger participants to exercise for mood regulation as both an emotional and meaningful present-focused goal. Those between 60 and 69 years of age were more likely to exercise for social contact as an emotionally meaningful goals and for weight loss as a present-focused goal. We recommend that exercises promoting both physical and mental health should be more popularized among younger adults.

Our study also showed that participants with an average level of education (high school/technical secondary school) were more likely to exercise for mood regulation than those with a lower or higher level of education. Similarly, in a behavior change intervention study, it was more difficult for groups with low and high levels of education and participants with mental diseases to adhere to exercise interventions than for others [40].

Jobs and mood disorders have generally been found to be correlated with each other [41–43]. Studies have shown that engaging in exercise served as a method of mood regulation to help people experience a positive mood for lengthier periods of time [44]. In our study, workers, administrative staff and professionals, and homemakers and retired individuals were more likely to exercise for mood regulation than students and business service employees. However, the job classification method of the questionnaire we used could not classify jobs involving engagement in high levels of physical activity, which reminded us that the results of our study should be interpreted with caution.

Physical inactivity and depression are involved in cause-and-effect relationships. Adults aged 18–64 years should perform at least 150 minutes of moderate-intensity aerobic physical activity throughout the week, at least 75 minutes of heavy-intensity aerobic physical activity throughout the week, or an equivalent combination of moderate- and heavy-intensity activity [45]. One-fourth of the European Union population did not meet the WHO recommendations for physical activity [46]. Depressed people were typically less active, while lower levels of physical activity increased the risk of depression [47]. It is well-known that engagement in regular physical activity is an important part of a healthy lifestyle. However, it was estimated that 60% of the United States population does not exercise regularly [48], and 63% of Canadians were not sufficiently active to obtain these health benefits [49]. Similarly, 44.9% (2355/5242) of participants in our study did not engage in physical exercise.

Exercise is a purpose-directed activity, and numerous investigations have studied individuals' reasons to exercise, such as health risks [50], treatment for depression [17], and social contact [38]. However, not all the exercise motivations were significantly related to physical activity because continuously maintaining a motivational attitude for a long period of time requires determination and can be quite challenging for many people, especially during this current busy daily life [51]. It was first expected that different exercise motivations would predict different physical practice frequencies, as various exercise motivations have been found to influence the effort expended during exercise [52]. Significant relationships were observed between mental health and both exercise frequency and duration [16]. The fact was mood regulation had no significant association with exercise frequency in our study, as did increasing physical activity, weight loss, and social contact. For the exercise motivation of disease prevention and treatment, participants were more likely to exercise less than once a week, once a week, or over four times a week than they were to exercise at other frequencies. With respect to entertainment, participants were more likely to exercise three times weekly and less likely to exercise over four times weekly than they were to engage in no exercise or exercise at other frequencies.

For exercise duration, a longer period of time is not necessarily better. Chekroud's study indicated that exercise duration between 30 min and 60 min (peaking at approximately 45 min) was associated with the lowest occurrence of mental health problems. A duration of more than 3 hours was associated with worse mental health [16]. However, in our study, exercise duration for each session or per week both showed no significant relationship with mood regulation. For the exercise motivation of disease prevention and treatment, participants were more likely to do exercise for less than 30 min or 30-60 min each session than they were to engage in no exercise or over 60 min of exercise each session; additionally, they prefer to exercise 0-30 min, 31-60 min, and 121-240 min per week than to engage in no exercise or other duration per week. For the motivation of social contact, fewer people would like to exercise for 30-60 min each session than to engage in no exercise or other duration of exercise each session. People who exercised for entertainment were more likely to exercise 61-120 min per week than to engage in no exercise or other duration per week. It was not surprising that participants who exercised to increase physical activity were less likely to exercise 0-30 min per week than they were to engage in no exercise or other duration per week.

Exercise motivations were found to have a strong relationship with exercise intensity [49]. Exercise of any intensity significantly regulated mood with no differential effect following mild-intensity, moderate-intensity, or heavy-intensity exercise [53]. Similarly, our research also showed no significant relationship between exercise intensity and mood regulation. A significant association was found between exercising for disease prevention and treatment and moderate and heavy exercise intensity. Some research has shown that heavy-intensity exercise can lead to health benefits above and beyond those offered by moderate-intensity exercise [54]. It was not surprising that participants exercising for the motivation of social contact were more likely to engage in mild-intensity exercise, sparing more energy for social activity. However, mild-intensity exercise showed no significant association with other exercise motivations, such as entertainment or weight loss.

Studies have shown that regular exercise is linked to the prevention of many chronic diseases, such as depression, type 2 diabetes, hypertension, obesity, and osteoporosis [55, 56]. However, changing exercise behaviors and maintaining the level of exercise required to reduce disease risk could be difficult to achieve, even when one is engaged in a lifestyle-change program [57]. Emotional problems played a key role in inactivity among individuals with chronic diseases [58, 59], but they showed no significant association between mood regulation and all kinds of diseases in our research. People with chronic diseases were more likely to be physically inactive, regardless of whether they had weak or strong intentions to exercise [60]. This might be the reason why fewer participants in our study would like to exercise for disease prevention and treatment with respect to hypertension, hyperlipidemia, hypercholesterolemia, osteoarthropathy, and cervical spondylopathy. Instead, participants preferred to exercise for increasing physical activity and weight loss. In a study of exercise motivation and weight loss among patients with hypertension, the majority reported being in the action stage or higher for weight loss [27].

For indexes 1 and 2, the compliance rates were very low. Only 16.64% (872/5242) were compliant with index 1, and 2.84% (149/5242) were compliant with index 2. One possible reason was that many patients with depression were physically inactive [61]. A study in Finland comprised 645 people and demonstrated that the risk of physical inactivity was more than twofold among persons with depressive symptoms than among nondepressed people [62]. In the Upper Bavarian Field Study, a representative community sample of 1,536 persons, people with depression were approximately three times more likely to be physically inactive than those who exercised regularly [63]. Another important result of our study was that higher education showed a significant association with reducing the mental burden and preventing depression. Participants who had a lower educational level were less likely to meet both indexes 1 and 2. This finding might be that the less-educated individuals have limited health consciousness and less knowledge about the advantages of physical activity than do more highly educated individuals [64]. The intervention study aiming to improve the level of education appeared successful in improving physical activity [65].

The limitations of our study should be considered. Firstly, our study was a cross-sectional design, and causal inferences cannot be made. Prospective study designs should be considered in further research. Secondly, it should be noted that this study did not investigate the status of depression. While this study did provide some insight into the link between exercise motivation and various sociodemographic characteristics, exercise behaviors, and physical conditions, the results must be interpreted with some degree of caution, as all of the exercise behavior measurements were provided via self-report. Thirdly, exercise measures were provided via self-reported in this study, and participants may overreport their frequencies or duration of exercise.

## 5. Conclusion

This study included six specific exercise motivations to identify the most important motivational forces behind sociodemographic characteristics and physical conditions and to understand motivation decisions leading to engagement in exercise of varying frequency, intensity, and durations. We also compared the differences between mood regulation and other exercise motivations and the possible influencing factors of exercise status in conjunction with mood regulation. Overall, the present investigation provides an important first step in determining the motivation profile of adults and older adults who exercise, which can be used as a reference to develop proper interventions in the future.

## Figures and Tables

**Table 1:** Characteristics of participants from Guangzhou with different exercise motivations.

Variables	Total (*n* = 5242)	Disease prevention and treatment ① (*n* = 2474, 47.2)	Entertainment ② (*n* = 2028, 36.7)	Mood regulation ③ (*n* = 1849, 35.3)	Increasing physical activity (*n* = 841, 16.0)	Weight loss (*n* = 811, 15.5)	Social contact (*n* = 438, 8.4)	① and ② (*n* = 781, 14.9)	① and ③ (*n* = 585, 11.2)	② and ③ (*n* = 546, 10.4)
Gender										
Male, *n* (%)	2480 (47.3)	1278 (51.7)	880 (43.4)	897 (48.5)	383 (45.5)	374 (46.1)	199 (45.4)	340 (43.5)	330 (56.4)	239 (43.8)
Female, *n* (%)	2762 (52.7)	1196 (48.3)	1148 (56.6)	952 (51.5)	458 (54.5)	437 (53.9)	239 (54.6)	441 (56.5)	255 (43.6)	307 (56.2)
*p* value		≤0.001	≤0.001	0.198	0.262	0.459	0.411	0.022	≤0.001	0.080
Age										
Mean ± SD	47.0 ± 14.0	41.5 ± 15.3	44.5 ± 9.8	48.5 ± 13.1	49.6 ± 14.1	52.3 ± 13.3	50.8 ± 13.1	42.6 ± 10.7	43.3 ± 17.5	45.8 ± 8.3
20-29, *n* (%)	863 (16.5)	800 (32.3)	150 (7.4)	249 (13.5)	124 (14.7)	75 (9.2)	35 (8.0)	95 (12.2)	227 (38.8)	22 (4.0)
30-39, *n* (%)	602 (11.5)	324 (13.1)	499 (24.6)	113 (6.1)	52 (6.2)	33 (4.1)	48 (11.0)	225 (28.8)	15 (2.6)	97 (17.8)
40-49, *n* (%)	1291 (24.6)	469 (19.0)	643 (31.7)	519 (28.1)	202 (24.0)	210 (25.9)	116 (26.5)	201 (25.7)	83 (14.2)	214 (39.2)
50-59, *n* (%)	1205 (23.0)	468 (18.9)	681 (33.6)	505 (27.3)	171 (20.3)	163 (20.1)	78 (17.8)	248 (31.8)	87 (14.9)	204 (37.4)
60-69, *n* (%)	1281 (24.4)	413 (16.7)	55 (2.7)	463 (25.0)	292 (34.7)	330 (40.7)	161 (36.8)	12 (1.5)	173 (29.6)	9 (1.6)
*p* value		≤0.001	≤0.001	≤0.001	≤0.001	≤0.001	≤0.001	≤0.001	≤0.001	≤0.001
Highest education level										
Primary or below, *n* (%)	881 (16.8)	315 (12.7)	272 (13.4)	309 (16.7)	173 (20.6)	171 (21.1)	96 (21.9)	91 (11.7)	83 (14.2)	90 (16.5)
Middle school, *n* (%)	1524 (29.1)	607 (24.5)	595 (29.3)	576 (31.2)	269 (32.0)	246 (30.3)	128 (29.2)	197 (25.2)	136 (23.2)	172 (31.5)
High/technical secondary school, *n* (%)	1249 (23.8)	613 (24.8)	447 (22.0)	485 (26.2)	185 (22.0)	201 (24.8)	96 (21.9)	183 (23.4)	168 (28.7)	113 (20.7)
College/junior college or above, *n* (%)	1588 (30.3)	939 (38.0)	714 (35.2)	479 (25.9)	214 (25.4)	193 (23.8)	118 (26.9)	310 (39.7)	198 (33.8)	171 (31.3)
*p* value		≤0.001	≤0.001	≤0.001	≤0.001	≤0.001	0.019	≤0.001	≤0.001	0.262
Job										
Students, *n* (%)	119 (2.3)	118 (4.8)	12 (0.6)	31 (1.7)	25 (3.0)	7 (0.9)	7 (1.6)	12 (1.5)	31 (5.3)	1 (0.2)
Administrative staff and professionals, *n* (%)	791 (15.1)	384 (15.5)	351 (17.3)	293 (15.8)	128 (15.2)	112 (13.8)	58 (13.2)	127 (16.3)	77 (13.2)	99 (18.1)
Business service employees, *n* (%)	968 (18.5)	542 (21.9)	546 (26.9)	277 (15.0)	121 (14.4)	104 (12.8)	73 (16.7)	237 (30.3)	93 (15.9)	131 (24.0)
Worker, *n* (%)	388 (7.4)	175 (7.1)	197 (9.7)	162 (8.8)	52 (6.2)	53 (6.5)	26 (5.9)	73 (9.3)	31 (5.3)	58 (10.6)
Others, *n* (%)	1029 (19.6)	544 (22.0)	471 (23.2)	389 (21.0)	121 (14.4)	137 (16.9)	75 (17.1)	174 (22.3)	130 (22.2)	129 (23.6)
Homemakers and retired individuals, *n* (%)	1947 (37.1)	711 (28.7)	451 (22.2)	697 (37.7)	394 (46.8)	398 (49.1)	199 (45.4)	158 (20.2)	223 (38.1)	128 (23.4)
*p* value		≤0.001	≤0.001	≤0.001	≤0.001	≤0.001	0.012	≤0.001	≤0.001	≤0.001
Exercise frequency										
No exercise	2355 (44.9)	1045 (42.2)	901 (44.4)	824 (44.6)	381 (45.3)	381 (47.0)	207 (47.3)	357 (45.7)	246 (42.1)	235 (43.0)
Less than once a week	373 (7.1)	195 (7.9)	156 (7.7)	127 (6.9)	46 (5.5)	53 (6.5)	29 (6.6)	63 (8.1)	42 (7.2)	40 (7.3)
Once a week	418 (8.0)	221 (8.9)	177 (8.7)	142 (7.7)	56 (6.7)	63 (7.8)	29 (6.6)	65 (8.3)	49 (8.4)	47 (8.6)
Twice a week	329 (6.3)	152 (6.1)	144 (7.1)	118 (6.4)	48 (5.7)	53 (6.5)	25 (5.7)	48 (6.1)	34 (5.8)	45 (8.2)
Three times a week	368 (7.0)	170 (6.9)	165 (8.1)	134 (7.2)	63 (7.5)	45 (5.5)	27 (6.2)	64 (8.2)	39 (6.7)	46 (8.4)
Four times a week	247 (4.7)	122 (4.9)	108 (5.3)	77 (4.2)	50 (5.9)	37 (4.6)	18 (4.1)	48 (6.1)	25 (4.3)	29 (5.3)
Over four times a week	1152 (22.0)	569 (23.0)	377 (18.6)	427 (23.1)	197 (23.4)	179 (22.1)	103 (23.5)	136 (17.4)	150 (25.6)	104 (19.0)
*p* value		0.003	≤0.001	0.631	0.087	0.607	0.748	0.014	0.425	0.166
Exercise duration each session										
No exercise	2355 (44.9)	1045 (42.2)	901 (44.4)	824 (44.6)	381 (45.3)	381 (47.0)	207 (47.3)	357 (45.7)	246 (42.1)	235 (43.0)
Less than 30 min	360 (6.9)	186 (7.5)	152 (7.5)	113 (6.1)	52 (6.2)	58 (7.2)	33 (7.5)	59 (7.6)	34 (5.8)	44 (8.1)
30-60 min	1522 (29.0)	761 (30.8)	624 (30.8)	550 (29.7)	220 (26.2)	217 (26.8)	102 (23.3)	233 (29.8)	181 (30.9)	176 (32.2)
Over 60 min	1005 (19.2)	482 (19.5)	351 (17.3)	362 (19.6)	188 (22.4)	155 (19.1)	96 (21.9)	132 (16.9)	124 (21.2)	91 (16.7)
*p* value		0.001	0.009	0.361	0.031	0.435	0.042	0.330	0.211	0.117
Exercise duration per week										
No exercise	2355 (44.9)	1045 (42.2)	901 (44.4)	824 (44.6)	381 (45.3)	381 (47.0)	207 (47.3)	357 (45.7)	246 (42.1)	235 (43.0)
<30 min	474 (9.0)	249 (10.1)	200 (9.9)	157 (8.5)	58 (6.9)	70 (8.6)	39 (8.9)	78 (10.0)	51 (8.7)	53 (9.7)
31-60 min	364 (6.9)	191 (7.7)	150 (7.4)	130 (7.0)	50 (5.9)	55 (6.8)	22 (5.0)	56 (7.2)	46 (7.9)	38 (7.0)
61-120 min	334 (6.4)	152 (6.1)	148 (7.3)	112 (6.1)	54 (6.4)	56 (6.9)	30 (6.8)	50 (6.4)	32 (5.5)	45 (8.2)
121-240 min	1115 (21.3)	553 (22.4)	442 (21.8)	401 (21.7)	190 (22.6)	152 (18.7)	79 (18.0)	171 (21.9)	133 (22.7)	127 (23.3)
>240 min	600 (11.4)	284 (11.5)	187 (9.2)	225 (12.2)	108 (12.8)	97 (12.0)	61 (13.9)	69 (8.8)	77 (13.2)	48 (8.8)
*p* value		0.001	≤0.001	0.692	0.105	0.460	0.144	0.241	0.382	0.109
Exercise intensity										
No exercise	2355 (44.9)	1045 (42.2)	901 (44.4)	824 (44.6)	381 (45.3)	381 (47.0)	207 (47.3)	357 (45.7)	246 (42.1)	235 (43.0)
Mild	676 (12.9)	304 (12.3)	248 (12.2)	227 (12.3)	119 (14.1)	104 (12.8)	78 (17.8)	93 (11.9)	76 (13.0)	76 (13.0)
Moderate	1505 (28.7)	743 (30.0)	606 (29.9)	543 (29.4)	241 (28.7)	219 (27.0)	105 (24.0)	222 (28.4)	177 (30.3)	177 (30.3)
Heavy	706 (13.5)	382 (15.4)	273 (13.5)	255 (13.8)	100 (11.9)	107 (13.2)	48 (11.0)	109 (14.0)	86 (14.7)	86 (14.7)
*p* value		≤0.001	0.407	0.663	0.376	0.587	0.001	0.799	0.474	0.022
BMI										
Mean ± SD	23.6 ± 3.3	23.3 ± 3.4	23.6 ± 3.3	23.7 ± 3.2	23.8 ± 3.2	23.7 ± 3.2	23.8 ± 3.1	23.4 ± 3.4	23.4 ± 3.2	23.9 ± 3.2
Underweight (<18.5 kg/m^2^), *n* (%)	230 (4.4)	143 (5.8)	82 (4.0)	70 (3.8)	33 (3.9)	26 (3.2)	17 (3.8)	45 (5.8)	31 (5.3)	12 (2.2)
Normal weight (≧18.5 to <23 kg/m^2^), *n* (%)	2110 (40.3)	1052 (42.5)	829 (40.9)	726 (39.2)	314 (37.3)	333 (41.1)	161 (36.8)	318 (40.7)	237 (40.5)	213 (39.1)
Overweight (≧23 to <25 kg/m^2^), *n* (%)	1322 (25.2)	628 (25.4)	484 (23.9)	477 (25.8)	215 (25.6)	195 (24.0)	125 (28.5)	196 (25.1)	155 (26.5)	132 (24.2)
Obese I (≧25 to <30 kg/m^2^), *n* (%)	1376 (26.2)	553 (22.3)	552 (27.2)	508 (27.5)	247 (29.4)	225 (27.7)	125 (28.5)	188 (24.1)	142 (24.3)	164 (30.0)
Obese II (≧30 kg/m^2^), *n* (%)	204 (3.9)	98 (4.0)	81 (4.0)	68 (3.7)	32 (3.8)	32 (4.0)	10 (2.4)	34 (4.3)	20 (3.4)	25 (4.5)
*p* value		≤0.001	0.412	0.269	0.179	0.355	0.133	0.248	0.554	0.050
Abdominal obesity										
Yes, *n* (%)	2238 (42.7)	1068 (43.2)	846 (41.7)	824 (44.6)	346 (41.1)	342 (42.1)	180 (41.1)	333 (42.6)	269 (45.9)	247 (45.3)
No, *n* (%)	3004 (57.3)	1406 (56.8)	1182 (58.3)	1025 (55.4)	495 (58.9)	469 (57.9)	258 (58.9)	448 (57.4)	316 (54.1)	299 (54.7)
*p* value		0.633	0.599	0.067	0.569	0.774	0.619	0.977	0.178	0.462
Basic disease										
Hypertension										
No, *n* (%)	4570 (87.2)	2219 (89.7)	1857 (91.6)	1609 (87.0)	708 (84.2)	667 (82.2)	375 (85.6)	712 (91.2)	500 (85.5)	507 (92.9)
Yes, *n* (%)	672 (12.8)	255 (10.3)	171 (8.4)	240 (13.0)	133 (15.8)	144 (17.8)	63 (14.4)	69 (8.8)	85 (14.5)	39 (7.1)
*p* value		≤0.001	≤0.001	0.798	0.005	≤0.001	0.306	≤0.001	0.189	≤0.001
Hyperlipidemia										
No, *n* (%)	4945 (94.3)	2353 (95.1)	1936 (95.5)	1755 (94.9)	776 (92.3)	764 (94.2)	418 (95.4)	742 (95.0)	551 (94.2)	532 (97.4)
Yes, *n* (%)	297 (5.7)	121 (4.9)	92 (4.5)	94 (5.1)	65 (7.7)	47 (5.8)	20 (4.6)	39 (5.0)	34 (5.8)	14 (2.6)
*p* value		0.022	0.005	0.179	0.005	0.862	0.298	0.378	0.871	0.001
Hypercholesterolemia										
No, *n* (%)	4970 (94.8)	2366 (95.6)	1928 (95.1)	1771 (95.8)	782 (93.0)	763 (94.1)	414 (94.5)	740 (94.8)	555 (94.9)	527 (96.5)
Yes, *n* (%)	272 (5.2)	108 (4.4)	100 (4.9)	78 (4.2)	59 (7.0)	48 (5.9)	24 (5.5)	41 (5.2)	30 (5.1)	19 (3.5)
*p* value		0.011	0.504	0.019	0.009	0.308	0.775	0.934	0.944	0.057
Diabetes										
No, *n* (%)	5088 (97.1)	2407 (97.3)	1988 (98.0)	1786 (96.6)	811 (96.4)	783 (96.5)	425 (97.0)	761 (97.4)	562 (96.1)	536 (98.2)
Yes, *n* (%)	154 (2.9)	67 (2.7)	40 (2.0)	63 (3.4)	30 (3.6)	28 (3.5)	13 (3.0)	20 (2.6)	23 (3.9)	10 (1.8)
*p* value		0.352	0.001	0.137	0.238	0.345	0.969	0.499	0.131	0.106
Coronary heart disease										
No, *n* (%)	5179 (98.8)	2449 (99.0)	2012 (99.2)	1832 (99.1)	828 (98.5)	799 (98.5)	426 (97.3)	772 (98.8)	580 (99.1)	543 (99.5)
Yes, *n* (%)	63 (1.2)	25 (1.0)	16 (0.8)	17 (0.9)	13 (1.5)	12 (1.5)	12 (2.7)	9 (1.2)	5 (0.9)	3 (0.5)
*p* value		0.229	0.029	0.166	0.318	0.430	0.002	0.891	0.414	0.139
Peptic ulcer										
No, *n* (%)	5138 (98.0)	2434 (98.4)	1991 (98.2)	1818 (98.3)	817 (97.1)	791 (97.5)	429 (97.9)	763 (97.7)	576 (98.5)	537 (98.4)
Yes, *n* (%)	104 (2.0)	40 (1.6)	37 (1.8)	31 (1.7)	24 (2.9)	20 (2.5)	9 (2.1)	18 (2.3)	9 (1.5)	9 (1.6)
*p* value		0.072	0.511	0.239	0.048	0.284	0.912	0.486	0.412	0.552
Osteoarthropathy										
No, *n* (%)	4887 (93.2)	2334 (94.3)	1921 (94.7)	1737 (93.9)	754 (89.7)	747 (92.1)	408 (93.2)	738 (94.5)	549 (93.8)	526 (96.3)
Yes, *n* (%)	355 (6.8)	140 (5.7)	107 (5.3)	112 (6.1)	87 (10.3)	64 (7.9)	30 (6.8)	43 (5.5)	36 (6.2)	20 (3.7)
*p* value		0.002	0.001	0.128	≤0.001	0.168	0.947	0.127	0.528	0.002
Cervical spondylopathy										
No, *n* (%)	4681 (89.3)	2243 (90.7)	1799 (88.7)	1656 (89.6)	721 (85.7)	730 (90.0)	393 (89.7)	696 (89.1)	519 (88.7)	488 (89.4)
Yes, *n* (%)	561 (10.7)	231 (9.3)	229 (11.3)	193 (10.4)	120 (14.3)	81 (10.0)	45 (10.3)	85 (10.9)	66 (11.3)	58 (10.6)
*p* value		0.003	0.272	0.648	≤0.001	0.474	0.762	0.859	0.630	0.949
Occupational disease										
No, *n* (%)	5166 (98.6)	2441 (98.7)	1994 (98.3)	1824 (98.6)	823 (97.9)	801 (98.8)	433 (98.9)	769 (98.5)	578 (98.8)	536 (98.2)
Yes, *n* (%)	76 (1.4)	33 (1.3)	34 (1.7)	25 (1.4)	18 (2.1)	10 (1.2)	5 (1.1)	12 (1.5)	7 (1.2)	10 (1.8)
*p* value		0.507	0.275	0.662	0.068	0.574	0.573	0.826	0.587	0.431

Note: a total of 5242 participants are involved in this study. As shown in the table, 47.2% of participants with exercise motivation of disease prevention and treatment coded as “①,” 36.7% of participants with exercise motivation of entertainment coded as “②,” 35.3% of participants with exercise motivation of mood regulation coded as “③,” 16.0% of participants with exercise motivation to increase physical activity, 15.5% of participants with exercise motivation to lose weight, 8.4% of participants with exercise motivation of social contact, and 14.9% of participants met ① and ②, 11.2% of participants met ① and ③, and 10.4% of participants met ② and ③. It is notable that data of participants who did not choose each of the exercise motivation above were shown in the table. Additionally, the questionnaire also contains exercise motivation of bodybuilding, increase exercise skill, unclear purpose, and others. Because the number of choosing these options was less than 5% of total participants, they were not listed in the table.

**Table 2:** Logistic regression models for exercise motivations.

Variables	Disease prevention and treatment ①	Entertainment ②	Mood regulation ③	Increasing physical activity	Weight loss	Social contact	① and ②	① and ③	② and ③
	OR (95% CI)	OR (95% CI)	OR (95% CI)	OR (95% CI)	OR (95% CI)	OR (95% CI)	OR (95% CI)	OR (95% CI)	OR (95% CI)
Gender (ref: male)									
Female	0.72 (0.64-0.80)	1.29 (1.16-1.45)	0.93 (0.83-1.04)	1.09 (0.94-1.26)	1.06 (0.91-1.23)	1.09 (0.89-1.32)	1.20 (1.03-1.39)	0.66 (0.56-0.79)	1.17 (0.98-1.40)
Age (ref: 20–29)									
30-39	0.09 (0.07-0.12)	23.03 (17.48-30.34)	0.57 (0.44-0.73)	0.56 (0.40-0.79)	0.61 (0.40-0.93)	2.05 (1.31-3.21)	4.83 (3.69-6.32)	0.07 (0.04-0.12)	7.34 (4.56-11.82)
40-49	0.05 (0.03-0.06)	4.72 (3.83-5.80)	1.66 (1.38-1.99)	1.11 (0.87-1.41)	2.04 (1.54-2.70)	2.34 (1.58-3.44)	1.49 (1.15-1.94)	0.19 (0.15-0.25)	7.60 (4.85-11.89)
50-59	0.05 (0.04-0.07)	6.18 (5.01-7.62)	1.78 (1.48-2.14)	0.99 (0.77-1.27)	1.64 (1.23-2.19)	1.64 (1.09-2.46)	2.10 (1.62-2.70)	0.22 (0.17-0.28)	7.79 (4.97-12.21)
60-69	0.04 (0.03-0.05)	0.21 (0.15-0.29)	1.40 (1.16-1.86)	1.76 (1.40-2.22)	3.65 (2.79-4.77)	3.40 (2.33-4.96)	0.08 (0.04-0.14)	0.44 (0.35-0.55)	0.27 (0.12-0.59)
Highest education level (ref: primary or below)									
Middle school	1.19 (1.00-1.41)	1.43 (1.20-1.71)	1.13 (0.95-1.34)	0.88 (0.71-1.08)	0.80 (0.64-0.99)	0.75 (0.57-0.99)	1.29 (0.99-1.68)	0.94 (0.71-1.26)	1.12 (0.85-1.46)
High/technical secondary school	1.73 (1.45-2.07)	1.24 (1.04-1.50)	1.18 (0.98-1.41)	0.71 (0.57-0.89)	0.88 (0.64-1.00)	0.68 (0.51-0.92)	1.49 (1.14-1.95)	1.49 (1.13-1.97)	0.87 (0.65-1.17)
College/junior college or above	2.60 (2.19-3.08)	1.83 (1.54-2.18)	0.80 (0.67-0.95)	0.64 (0.51-0.79)	0.57 (0.46-0.72)	0.66 (0.50-0.87)	2.11 (1.64-2.70)	1.37 (1.05-1.80)	1.06 (0.81-1.39)
Job (ref: students)									
Administrative staff and professionals	0.01 (0.00-0.06)	7.11 (3.85-13.13)	1.67 (1.08-2.58)	0.73 (0.45-1.17)	2.64 (1.20-5.81)	1.27 (0.56-2.84)	1.71 (0.91-3.19)	0.31 (0.19-0.49)	8.30 (1.15-59.89)
Business service employees	0.01 (0.00-0.08)	11.54 (6.27-21.23)	1.14 (0.74-1.75)	0.54 (0.33-0.87)	1.93 (0.87-4.25)	1.31 (0.59-2.90)	2.89 (1.56-5.34)	0.30 (0.19-0.48)	16.91 (2.34-122.05)
Worker	0.01 (0.00-0.05)	9.20 (4.90-17.25)	2.04 (1.29-3.21)	0.58 (0.34-0.99)	2.53 (1.12-5.73)	1.15 (0.49-2.72)	2.07 (1.08-3.95)	0.25 (0.14-0.43)	20.73 (2.84-151.33)
Others	0.01 (0.00-0.07)	7.53 (4.09-13.84)	1.73 (1.12-2.65)	0.50 (0.31-0.81)	2.46 (1.12-5.39)	1.26 (0.57-2.80)	1.82 (0.98-3.37)	0.41 (0.26-0.64)	18.46 (2.56-133.27)
Homemakers and retired individuals	0.01 (0.00-0.04)	2.69 (1.47-4.93)	1.58 (1.04-2.41)	0.95 (0.61-1.50)	4.11 (1.90-8.89)	1.82 (0.84-3.96)	0.79 (0.42-1.46)	0.37 (0.24-0.57)	16.88 (2.33-122.14)
Exercise frequency (ref: no exercise)									
Less than once a week	1.37 (1.10-1.71)	1.16 (0.93-1.45)	0.96 (0.76-1.21)	0.73 (0.53-1.01)	0.86 (0.63-1.17)	0.88 (0.58-1.31)	1.14 (0.85-1.53)	1.09 (0.77-1.54)	1.08 (0.76-1.55)
Once a week	1.41 (1.14-1.73)	1.19 (0.96-1.46)	0.96 (0.77-1.19)	0.80 (0.59-1.08)	0.92 (0.69-1.23)	0.77 (0.52-1.16)	1.03 (0.77-1.37)	1.14 (0.82-1.58)	1.14 (0.82-1.59)
Twice a week	1.08 (0.85-1.36)	1.26 (1.00-1.59)	1.04 (0.82-1.32)	0.89 (0.64-1.23)	1.00 (0.73-1.36)	0.85 (0.55-1.31)	0.96 (0.69-1.33)	0.99 (0.68-1.44)	1.43 (1.02-2.01)
Three times a week	1.08 (0.86-1.34)	1.31 (1.05-1.64)	1.06 (0.85-1.34)	1.07 (0.80-1.43)	0.72 (0.52-1.01)	0.82 (0.54-1.25)	1.18 (0.88-1.58)	1.02 (0.71-1.45)	1.29 (0.92-1.81)
Four times a week	1.22 (0.94-1.59)	1.25 (0.96-1.63)	0.84 (0.64-1.12)	1.32 (0.95-1.83)	0.91 (0.63-1.32)	0.82 (0.49-1.35)	1.35 (0.97-1.89)	0.97 (0.63-1.49)	1.20 (0.80-1.81)
Over four times a week	1.22 (1.06-1.41)	0.79 (0.68-0.91)	1.09 (0.95-1.27)	1.07 (0.89-1.29)	0.95 (0.79-1.16)	1.02 (0.80-1.31)	0.75 (0.61-0.93)	1.28 (1.03-1.59)	0.90 (0.70-1.14)
Exercise duration each session (ref: no exercise)									
Less than 30 min	1.34 (1.07-1.67)	1.18 (0.94-1.48)	0.85 (0.67-1.08)	0.88 (0.64-1.20)	1.00 (0.74-1.35)	1.05 (0.71-1.54)	1.10 (0.81-1.48)	0.89 (0.61-1.30)	1.26 (0.89-1.77)
30-60 min	1.25 (1.10-1.43)	1.12 (0.98-1.28)	1.05 (0.92-1.20)	0.88 (0.73-1.05)	0.86 (0.72-1.03)	0.75 (0.58-0.95)	1.01 (0.85-1.21)	1.16 (0.94-1.42)	1.18 (0.96-1.45)
Over 60 min	1.16 (1.00-1.34)	0.87 (0.74-1.01)	1.05 (0.90-1.22)	1.19 (0.98-1.45)	0.95 (0.77-1.16)	1.10 (0.85-1.41)	0.85 (0.68-1.05)	1.21 (0.96-1.52)	0.90 (0.70-1.16)
Exercise duration per week (ref: no exercise)									
<30 min	1.39 (1.14-1.69)	1.18 (0.96-1.44)	0.92 (0.75-1.13)	0.72 (0.54-0.97)	0.90 (0.68-1.18)	0.93 (0.65-1.33)	1.10 (0.84-1.44)	1.03 (0.75-1.42)	1.14 (0.83-1.56)
31-60 min	1.38 (1.11-1.73)	1.13 (0.90-1.42)	1.03 (0.82-1.30)	0.83 (0.60-1.13)	0.92 (0.68-1.25)	0.67 (0.42-1.05)	1.02 (0.75-1.38)	1.24 (0.89-1.74)	1.05 (0.73-1.51)
61-120 min	1.05 (0.83-1.32)	1.28 (1.02-1.63)	0.94 (0.74-1.20)	1.00 (0.73-1.36)	1.04 (0.77-1.42)	1.02 (0.69-1.53)	0.99 (0.72-1.36)	0.91 (0.62-1.34)	1.41 (1.00-1.98)
121-240 min	1.23 (1.07-1.42)	1.06 (0.92-1.23)	1.04 (0.90-1.21)	1.06 (0.88-1.29)	0.82 (0.67-1.00)	0.79 (0.60-1.04)	1.01 (0.83-1.24)	1.16 (0.93-1.45)	1.16 (0.92-1.46)
>240 min	1.13 (0.95-1.35)	0.73 (0.60-0.89)	1.12 (0.93-1.34)	1.14 (0.90-1.44)	1.00 (0.78-1.28)	1.17 (0.87-1.59)	0.73 (0.55-0.96)	1.26 (0.96-1.66)	0.79 (0.57-1.09)
Exercise intensity (ref: no exercise)									
Light	1.02 (0.86-1.22)	0.94 (0.78-1.12)	0.94 (0.78-1.13)	1.11 (0.88-1.39)	1.11 (0.88-1.39)	1.35 (1.03-1.78)	0.89 (0.70-1.14)	1.09 (0.83-1.43)	0.82 (0.60-1.11)
Medium	1.22 (1.07-1.39)	1.09 (0.95-1.24)	1.05 (0.92-1.20)	0.99 (0.83-1.18)	0.99 (0.83-1.18)	0.78 (0.61-0.99)	0.97 (0.81-1.16)	1.14 (0.93-1.40)	1.26 (1.03-1.55)
Heavy	1.48 (1.25-1.75)	1.02 (0.86-1.21)	1.05 (0.88-1.25)	0.86 (0.67-1.09)	0.86 (0.67-1.09)	0.76 (0.55-1.05)	1.02 (0.81-1.29)	1.19 (0.92-1.54)	0.99 (0.75-1.32)
BMI (ref: underweight)									
Normal weight (≧18.5 to <23 kg/m^2^)	0.56 (0.38-0.83)	1.19 (0.81-1.75)	1.14 (0.76-1.71)	1.11 (0.66-1.88)	1.46 (0.84-2.54)	0.65 (0.29-1.45)	0.82 (0.50-1.34)	0.70 (0.38-1.27)	2.54 (1.24-5.19)
Overweight (≧23 to <25 kg/m^2^)	0.41 (0.31-0.55)	1.21 (0.90-1.62)	1.34 (0.99-1.81)	1.31 (0.88-1.94)	1.53 (1.00-2.36)	1.25 (0.74-2.12)	0.65 (0.45-0.93)	0.74 (0.49-1.12)	2.46 (1.34-4.50)
Obese I (≧25 to <30 kg/m^2^)	0.55 (0.41-0.73)	1.04 (0.78-1.40)	1.29 (0.95-1.75)	1.16 (0.78-1.72)	1.36 (0.88-2.10)	1.31 (0.77-2.22)	0.72 (0.50-1.03)	0.85 (0.56-1.29)	2.02 (1.10-3.70)
Obese II (≧30 kg/m^2^)	0.61 (0.46-0.80)	1.17 (0.88-1.55)	1.20 (0.89-1.61)	1.04 (0.71-1.54)	1.47 (0.96-2.25)	1.04 (0.62-1.74)	0.73 (0.52-1.03)	0.81 (0.54-1.21)	2.04 (1.12-3.71)
Basic disease									
Hypertension (ref: no hypertension)									
Yes	0.65 (0.55-0.77)	0.50 (0.42-0.60)	1.02 (0.86-1.21)	1.35 (1.10-1.65)	1.60 (1.30-1.95)	1.16 (0.88-1.53)	0.62 (0.48-0.81)	1.18 (0.92-1.51)	0.49 (0.35-0.69)
Hyperlipidemia (ref: no hyperlipidemia)									
Yes	0.76 (0.60-0.96)	0.70 (0.54-0.90)	0.84 (0.66-1.08)	1.51 (1.13-2.00)	1.03 (0.75-1.42)	0.78 (0.49-1.25)	0.86 (0.61-1.21)	1.03 (0.71-1.49)	0.41 (0.24-0.71)
Hypercholesterolemia (ref: no hypercholesterolemia)									
Yes	0.73 (0.57-0.93)	0.92 (0.71-1.18)	0.73 (0.56-0.95)	1.48 (1.10-2.00)	1.18 (0.86-1.63)	1.07 (0.69-1.64)	1.02 (0.72-1.43)	0.99 (0.67-1.46)	0.63 (0.39-1.02)
Diabetes (ref: no diabetes)									
Yes	0.86 (0.62-1.19)	0.55 (0.38-0.79)	1.28 (0.92-1.77)	1.28 (0.85-1.92)	1.22 (0.81-1.85)	1.01 (0.57-1.80)	0.85 (0.53-1.37)	1.42 (0.90-2.22)	0.59 (0.31-1.13)
Coronary heart disease (ref: no coronary heart disease)									
Yes	0.73 (0.44-1.22)	0.54 (0.30-0.95)	0.68 (0.39-1.18)	1.37 (0.74-2.53)	1.29 (0.69-2.43)	2.63 (1.39-4.97)	0.95 (0.47-1.94)	0.68 (0.27-1.71)	0.43 (0.13-1.37)
Osteoarthropathy (ref: no osteoarthropathy)									
Yes	0.71 (0.57-0.89)	0.67 (0.53-0.84)	0.84 (0.66-1.05)	1.78 (1.38-2.29)	1.22 (0.92-1.62)	1.01 (0.69-1.49)	0.78 (0.56-1.08)	0.89 (0.63-1.27)	0.50 (0.31-0.78)
Cervical spondylopathy (ref: no cervical spondylopathy)									
Yes	0.76 (0.64-0.91)	1.11 (0.92-1.32)	0.96 (0.80-1.15)	1.50 (1.20-1.86)	0.91 (0.71-1.17)	0.95 (0.69-1.31)	1.02 (0.80-1.31)	1.07 (0.81-1.40)	0.99 (0.74-1.32)

**Table 3:** Comparison of the characteristics of the adults and senior adults from Guangzhou with exercise indexes that is good for mental health.

Variables	Index 1					Index 2				
	Meet (*n* = 872)		Unmet (*n* = 4370)		*p* value	Meet (*n* = 149)		Unmet (*n* = 5093)		*p* value
	*n*	%	*n*	%		*n*	%	*n*	%	
Gender					0.627					0.114
Male	406	46.6	2074	47.5		80	53.7	2400	47.1	
Female	466	53.4	2296	52.5		69	46.3	2693	52.9	
Age					0.009					0.138
20-29	169	19.4	694	15.9		20	13.4	843	16.6	
30-39	110	12.6	492	11.3		15	10.1	587	11.5	
40-49	206	23.6	1085	24.8		50	33.6	1241	24.4	
50-59	168	19.3	1037	23.7		33	22.1	1172	23.0	
60-69	219	25.1	1062	24.3		31	20.8	1250	24.5	
Highest education level					<0.001					0.001
Primary or below	107	12.3	774	17.7		13	8.7	868	17.0	
Middle school	219	25.1	1305	29.9		34	22.8	1490	29.3	
High/technical secondary school	233	26.7	1016	23.2		37	24.8	1212	23.8	
College/junior college or above	313	35.9	1275	29.2		65	43.6	1523	29.9	
Job					0.001					0.093
Students	20	2.3	99	2.3		2	1.3	117	2.3	
Administrative staff and professionals	128	14.7	663	15.2		35	23.5	756	14.8	
Business service employees	144	16.5	824	18.9		27	18.1	941	18.5	
Worker	45	5.2	343	7.8		11	7.4	377	7.4	
Others	214	24.5	815	18.6		28	18.8	1001	19.7	
Homemakers and retired individuals	321	36.8	1626	37.2		46	30.9	1901	37.3	
BMI					0.088					0.292
Underweight (<18.5 kg/m^2^)	24	2.8	206	4.7		4	2.7	225	4.4	
Normal weight (≧18.5 to <23 kg/m^2^)	362	41.5	1749	40.0		66	44.3	2045	40.2	
Overweight (≧23 to <25 kg/m^2^)	210	24.1	1112	25.4		36	24.2	1286	25.3	
Obese I (≧25 to <30 kg/m^2^)	242	27.8	1133	25.9		42	28.2	1334	26.2	
Obese II (≧30 kg/m^2^)	34	3.9	170	3.9		1	0.7	203	4.0	
Abdominal obesity					0.907					0.259
Yes	374	42.9	1862	42.6		55	36.9	2184	42.9	
No	498	57.1	2508	57.4		94	63.1	2909	57.1	
Basic disease										
Hypertension					0.981					0.129
No	760	87.2	3810	87.2		136	91.3	4434	87.1	
Yes	112	12.8	560	12.8		13	8.7	659	12.9	
Hyperlipidemia					0.124					0.920
No	813	93.2	4132	94.6		142	95.3	4803	94.3	
Yes	59	6.8	238	5.4		7	4.7	290	5.7	
Hypercholesterolemia					0.900					0.498
No	826	94.7	4144	94.8		141	94.6	4829	94.8	
Yes	46	5.3	226	5.2		8	5.4	264	5.2	
Diabetes					0.336					0.172
No	842	96.6	4246	97.2		146	98.0	5030	98.8	
Yes	30	3.4	124	2.8		3	2.0	63	1.2	
Coronary heart disease					0.391					0.534
No	859	98.5	4320	98.9		149	100.0	4993	98.0	
Yes	13	1.5	50	1.1		0	0.0	100	2.0	
Peptic ulcer					0.130					0.534
No	849	97.4	4289	98.1		145	97.3	4993	98.0	
Yes	23	2.6	81	1.9		4	2.7	100	2.0	
Osteoarthropathy					0.380					0.764
No	807	92.5	4080	93.4		138	92.6	4749	93.2	
Yes	65	7.5	290	6.6		11	7.4	344	6.8	
Cervical spondylopathy					0.128					0.777
No	766	87.8	3915	89.6		132	88.6	4549	89.3	
Yes	106	12.2	455	10.4		17	11.4	544	10.7	

Note: index 1 means exercise 30-60 min each session and 3-5times per week or over; index 2 means exercise purpose is mood regulation and exercise 60-120 min each week.

**Table 4:** Logistic regression models for exercise indexes.

Variables	Index 1	Index 2
	OR (95% CI)	OR (95% CI)
Gender (ref: male)		
Female	1.04 (0.90-1.20)	0.77 (0.55-1.07)
Age (ref: 20–29)		
30-39	1.05 (0.52-2.11)	0.95 (0.72-1.25)
40-49	2.04 (1.16-3.59)	0.90 (0.70-1.15)
50-59	1.72 (0.92-3.22)	0.82 (0.63-1.07)
60-69	1.77 (0.79-3.96)	1.05 (0.76-1.46)
Highest education level (ref: primary or below)		
Middle school	1.49 (0.77-2.87)	1.30 (1.00-1.67)
High/technical secondary school	2.13 (1.10-4.10)	1.76 (1.36-2.28)
College/junior college or above	3.41 (1.74-6.66)	2.08 (1.58-2.75)
Job (ref: students)		
Administrative staff and professionals	2.20 (0.49-9.95)	1.18 (0.69-2.04)
Business service employees	1.59 (0.35-7.21)	1.05 (0.62-1.80)
Worker	2.18 (0.43-11.02)	1.12 (0.60-2.08)
Others	1.89 (0.42-8.55)	1.81 (1.06-3.08)
Homemakers and retired individuals	1.77 (0.36-8.69)	1.42 (0.80-2.52)

## Data Availability

The data used to support the findings of this study are available from the corresponding author upon request.
